# Survival of Neural Stem Cells Undergoing DNA Damage-Induced Astrocytic Differentiation in Self-Renewal-Promoting Conditions *In Vitro*

**DOI:** 10.1371/journal.pone.0087228

**Published:** 2014-01-27

**Authors:** Leonid Schneider

**Affiliations:** 1 IFOM Foundation - The FIRC Institute of Molecular Oncology Foundation, Milan, Italy; 2 Fachbereich Biologie, Technische Universität Darmstadt, Darmstadt, Germany; University of Nebraska Medical Center, United States of America

## Abstract

We recently reported that neural stem cells (NSCs) become senescent and commit to astrocytic differentiation upon X-ray irradiation. Surprisingly, under self-renewing culture conditions, some of these senescent cells undergo *p53*-independent apoptosis, which can be suppressed by caspase inhibition and *BCL2* overexpression. Inhibition of apoptosis proved beneficial for astroglial differentiation efficiency; hence the toxicity of DNA damage on NSCs was specifically tested in context of the culture conditions. In this regard, self-renewal-promoting culture conditions proved incompatible with terminal astrocyte differentiation and impacted negatively on the viability of NSCs following DNA damage-induced cell cycle exit. On the contrary, a switch to differentiation-supporting conditions ablated apoptosis and conveyed tolerance to DNA damage. Thus, stem cell death has likely not originated from DNA break toxicity, while the potentially confounding effect of stem cell niche should always be taken in consideration in stem cell irradiation experiments.

## Introduction

DNA double strand breaks, e.g. induced by ionizing irradiation, are the most toxic damage to eukaryotic genome and can rapidly result in apoptosis or permanent cell cycle exit, i.e., cellular senescence, both mediated by DNA damage response (DDR) signaling factors [1], [2], most prominently p53 [3]. Senescent cells commonly retain their viability despite residual DNA damage and become resistant to apoptosis [1]. Understanding physiological responses of somatic stem cells to DNA damage is imperative in the context of tissue homeostasis, organismal ageing and tumorigenesis. Neural stem cells (NSCs) can be derived from brain tissues or pluripotent stem cells and cultured *in vitro* in defined serum-free conditions, which promote their self-renewal by suppressing differentiation and stimulating proliferation [4], [5]. We demonstrated that, following irradiation-induced cellular senescence, NSCs rapidly lose expression of self-renewal markers such as Nestin and undergo astrocytic differentiation, associated with upregulation of the typical filament GFAP, while the latter relied on senescence-associated secretion of BMP2 and was boosted by absence of the *p53* gene [6]. Similarly to terminally differentiated astrocytes, these NSCs also transcriptionally downregulate genes of DNA damage response (DDR) cascade such as ATM and p53, while retaining the capacity for double strand break repair [6], [7]. Yet despite inefficient DDR signaling, a loss of viability was observed in irradiated NSC cultures, which mechanistic origins in regard to DNA damage per se and astroglial differentiation were elucidated in this study.

## Materials and Methods

### Cell culture

Murine ES-derived NSCs of E14Tg2a ES-background and other wildtype and *p53-/-* NSCs [6] were grown in Euromed-N cell culture medium (Euroclone), supplemented with L-Glutamine and Penicillin/Streptomycin, 1× N2 supplement (Invitrogen) and 20 ng/ml each murine EGF and FGF2 (ProSpec, Israel). For medium modifications, caspase inhibitor Q-VD-OPH (SM Biochemicals), BMP2 (ProSpec, Israel) or fetal calf serum (FCS) were added at 10 µM or 20 ng/ml or 10%, respectively. For neuronal differentiation, cells seeded on 3 µg/ml Laminin were switched to modified medium as in [8]: Euromed-N (Euroclone)/Neurobasal (Invitrogen) 1∶3, 0.5× N2 and 1.5× B27 supplement (Invitrogen), 10 ng FGF2 and 20 ng BDNF (ProSpec, Israel). For *BCL2* overexpression, a retroviral pBABE-puro vector carrying human *BCL2* cDNA (Addgene, plasmid 21144) or empty pBABE-puro vector were transfected into ecotropic 293T Phoenix cells using calcium-phosphate method. NSC at ∼30% confluence were then infected with viral supernatants, supplemented with 8 µg/ml polybrene (Sigma Aldrich) and selected 24 h later with 0.5 µg/ml puromycine (Sigma Aldrich) until no cell death was visually detectable and irradiated.

### X-ray irradiations

X-ray irradiation of cells was performed in a Faxitron RX-650 device at ∼2 Gy/min for 5 min and on GE Isovolt Titan E device at 2.8 Gy/min for 3.4 min; both total of 10 Gy. Cells were not passaged after irradiation and medium change was performed on day 1 after and then every other day.

### Apoptosis assays

For MTT (3-(4,5-Dimethylthiazol-2-yl)-2,5-diphenyltetrazolium bromide) survival assay, cells on 96well plates in quadruplicates were incubated for 1.5 h at 37°C with 0.5 mg/ml MTT (Sigma Aldrich) in phenol red-free DMEM medium (Invitrogen). Formazan crystals were dissolved by stop solution (0.04 M HCl in isopropanol), absorbance measured at 570 nm with background subtraction at 650 nm. For flow cytometrical (FACS) apoptosis assays, cells were fixed in 75% ethanol and stained with propidium iodide (Sigma Aldrich) to measure Sub-G_1_ DNA content; for TUNEL assay cells were first treated with “In Situ Cell Death Detection Kit, Fluorescein” (Roche), according to manufacturer's instructions. FACS acquisition and analysis were performed in experimental triplicates on BD FACScalibur using CellQuest software.

### Microarray analysis

The excerpts from microarray gene expression data refer to analysis of non-irradiated and irradiated NSCs at d7 in quadruplicates, originally published in [6], which raw data is openly available in the GEO database with accession number GSE38031.

### Immunostainings

For western blotting, cells were lysed in NP40 lysis buffer (1% NP40, 50 mM Tris-Cl pH 8, 150 mM NaCl, 2 mM EDTA, 1 mM DTT, 1 mM NaF, 100 µM Na_2_VO_4_ and protease inhibitor cocktail (Roche), resolved by SDS-PAGE, transferred to nitrocellulose membranes (Protran) and probed with primary antibodies: cleaved Caspase-3 (Asp175, Cell Signaling, #9664), BCL2 (Santa Cruz, #sc-7382), Nestin (#611658, BD Biosciences), GFAP (#Z0334 Dako), α-tubulin (#T6199, Sigma Aldrich), Vinculin (#V4505, Sigma Aldrich). HRP-coupled secondary antibodies (Sigma Aldrich) and ECL Plus™ Western Blotting Detection Reagents and X-ray films (Amersham) were used for signal detection.

For wide-field immunofluorescence microscopy, cells on glass cover slips were fixed in 4% paraformaldehyde and permeabilized with 0.2% Triton X100. After blocking and antibody staining in 0.5% BSA/0.2% gelatin in PBS (secondary antibody AlexaFluor 488-labeled, Invitrogen), nuclear DNA was stained by DAPI (Sigma Aldrich).

### Gene expression analysis

Total RNA was extracted from live cells with Trizol reagent (Invitrogen). 1 µg of total RNA was used for retrotranscription using VILO reverse transcription kit (Invitrogen) and estimated 20 ng of cDNA in 25 µl reaction volume were analyzed in triplicate by quantitative RT-PCR amplification on a Light Cycler 480 system (Roche) using SYBR Green assay (QuantiFast SYBR Green PCR Kit, Qiagen), all according to manufacturer's instructions. CT-values were obtained by calculation of the second derivative using Light Cycler 480 software and normalized among samples against a housekeeping gene *β-2-microglobulin* (*B2M*). RT-minus preparations (without reverse transcriptase enzyme) proved to be negative. Following forward and reverse primers (FP and RP) were designed with Roche UniversalProbe Library online software against *Mus musculus*:

*ATM*: FP: TGCAGATTTATATCCATCATCCAC; RP: TTTCATGGATTCATAAGCACCTT

*B2M*: FP: CTGCAGAGTTAAGCATGCCAGTA; RP: TCACATGTCTCGATCCCAGTAGA

*BAX*: FP: GTGAGCGGCTGCTTGTCT; RP: GGTCCCGAAGTAGGAGAGGA

*gfap*: FP: tggaggaggagatccagttc; RP: agctgctcccggagttct

*Ki67*: FP: GCTGTCCTCAAGACAATCATCA; RP: GGCGTTATCCCAGGAGACT

*Nestin*: FP: ctgcaggccactgaaaagtt; RP: tctgactctgtagaccctgcttc

*PUMA*: FP: TTCTCCGGAGTGTTCATGC; RP: TACAGCGGAGGGCATCAG

*S100β*: FP: AACAACGAGCTCTCTCACTTCC; RP: CTCCATCACTTTGTCCACCA

*tUJ1*: FP: gcgcatcagcgtatactacaa; RP: catggttccaggttccaagt

*mbp*: FP: ggcacgctttccaaaatct; RP: ccatgggagatccagagc

## Results and Discussion

We have recently reported that terminally differentiated NSC-derived astrocytes are apoptosis-resistant following ionizing irradiation [7]. Their parental self-renewing NSCs, respond to irradiation by a senescent-like cell cycle exit and astroglial differentiation, associated with transcriptional attenuation of DDR signaling and foci formation [6]. However, we also observed a degree of cell death in irradiated NSCs (Fig. 1A), which was however delayed (Fig. 1B) and occurring in cells progressively undergoing senescence and differentiation (∼80% resp. ∼50% at day 3 [6]). Microarray analysis of irradiated NSCs showed that this apoptotic cell death was associated with upregulated pro-apoptotic genes like *PUMA* (associated with p53-dependent and p53-independent apoptosis [9], also in NSC [10]), and to a lesser extent, *BAX, BID, APAF1* and *Caspase-3* and -*9* (Fig. 1C). Indeed, the delayed cell death in irradiated NSC does apparently follow the canonical caspase-dependent mechanism, since the pharmacological caspase inhibitor Q-VD-OPH was effective in suppressing the radiation-induced cell death (Fig. 1D). Peculiarly though, key anti-apoptotic genes like *XIAP, BCL2* and *BCL-XL* were found upregulated and apical apoptosis inducers *ATM* and *p53* downregulated in irradiated NSCs (Fig. 1C and [6]). Even more strikingly, genetic *p53*-deficiency did not reduce apoptosis in irradiated NSCs, as would be expected [3], but in fact resulted in a significantly higher cell death rate compared to wild types (Fig. 1E), associated with a rather prominent presence of active caspase-3, as it featured above the assay detection threshold in irradiated p53-/- cells (Fig. 1F). Moreover, not only irradiation-induced apoptosis in NSCs proved p53-independent, irradiated *p53-/-* NSCs exited cell cycle just as isogenic wild type cells (>80% at d3), directly correlating with the more pronounced astroglial differentiation of the former [6]. As irradiated and differentiating NSCs were cultured in self-renewal-promoting conditions, we suggest that their increased apoptosis must be causally connected to their increased differentiation under such unfavorable culture conditions.

**Figure 1:** NSC undergo a delayed and p53-independent apoptosis upon irradiation. (A)NSC cell density before (T0, normalized b as 100%) and after irradiation as measured by colorimetric MTT assay. Error bars: SD. (B)Apoptosis analysis by flow cytometrical TUNEL assay on non-irradiated (non-irr) NSCs and following irradiation. Error bars: SD. (C)Expression changes in apoptosis-relevant genes in NSCs at day 7 after irradiation compared to non-irradiated NSCs, based on microarray dataset originally published in [6]. (D)Flow cytometry analysis for apoptosis-associated DNA fragmentation (Sub-G1) of irradiated NSCs treated with pan-caspase inhibitor Q-VD-OPH (10 µM). Error bars: SD. (E)Flow cytometry analysis for apoptosis-associated DNA fragmentation (Sub-G1) of irradiated p53-deficient and isogenic wild type NSC. Error bars: SD. (F)Western blot analysis of irradiated p53-deficient and isogenic wild type NSC for apoptosis-associated appearance of active caspase 3. Loading control: α-tubulin.

Given a possible role of *BCL2* in NSCs' radiation response (Fig. 1C), an overexpression of this anti-apoptotic gene in irradiated NSCs lead to an efficient reduction in their apoptotic response (Fig. 2A). With such reduced apoptotic signalling, *BCL2*-overexpressing cells proved qualitatively more committed to irradiation-induced astrocytic differentiation, by downregulating Nestin and upregulating not only GFAP, but also the more mature astrocyte marker *S100β* [6], [11] (Fig. 2B,C). At the same time, despite some bias of *BCL2*-overexpressing cells towards glial fate, no clear evidence of neuronal or oligodendrocyte differentiation was detected in either vector- or *BCL2*-transduced and irradiated NSCs (Fig. 2D). These data, together with the reduced viability of *p53-/-* NSCs, suggest that apoptotic stimuli may be somehow connected to the ongoing DNA damage-induced astroglial differentiation of irradiated NSCs.

**Figure 2:** Inhibition of apoptosis in irradiated NSCs by *BCL2*-overexpression allows a more efficient astroglial differentiation. (A)Vector-transduced or *BCL2*-overexpressing NSC were irradiated, apoptotic cell death analyzed by TUNEL assay. Error bars: SD. (B)Gene expression analysis at day 3 post irradiation of vector-transduced or *BCL2*-overexpressing NSC for the expression of stem cell marker *Nestin*, astrocyte markers *GFAP* and *S100β*, pro-apoptotic genes *BAX* and *PUMA*, normalized against respective non-irr cells. Technical triplicates, error bars: SD. (C)Western blot analysis of vector-transduced or *BCL2*-overexpressing NSC for expression of Nestin and GFAP following irradiation. Loading control: vinculin. (D)Gene expression analysis as in (A) for the expression of markers of mature neurons (*TUJ1/β-tubulinIII*) and oligodendrocytes (*MBP*), normalized against respective non-irr cells. Cave: both gene products were detected at rather low expression levels (high qPCR-cycle number). Technical triplicates, error bars: SD.

To investigate the possible impact of culture conditions on the viability of irradiated NSCs in context of DNA-damage induced astroglial differentiation, NSCs were seeded on laminin and transferred to neuronal differentiation medium immediately after irradiation. This treatment, though promoting highly efficient neuronal differentiation of irradiated NSCs [6], also lead to a significantly higher fraction of apoptotic cells (Fig. 3A). This may indicate a possible conflict between cell-autologous astroglial fate determination and neuronal differentiation stimuli from the culture. On the other hand, supplementing the self-renewal medium with BMP2, which we recently reported to play a key role in induction of astroglial differentiation in irradiated NSCs [6], was not sufficient to confer any detectable viability benefit (Fig. 3A).

**Figure 3:** Apoptosis in irradiated NSC is dependent on culture conditions. (A)Flow cytometry analysis for apoptosis-associated DNA fragmentation (Sub-G1) of irradiated NSCs, cultured in standard self-renewal medium, or supplemented with BMP2 (20 ng/ml), or switched to BDNF-containing Neuronal differentiation medium. Error bars: SD. (B)Representative immunofluorescence analysis of GFAP expression in non-irr and irr NSC subjected for 24 h to FCS. DNA was stained with DAPI. Magnification: 40×. (C)Gene expression analysis of astrocytes derived by 10% FCS from NSC (FCS d3), and when switched back to NSC culture medium, normalized against self-renewing NSC. Technical triplicates, error bars: SD. (D)TUNEL assay for irradiated NSC at day 3, cultured in unmodified (self-renewal promoting) medium or supplemented with FCS (astroglial differentiation medium), either immediately (d0+3) or 24 h after irr (d1+2). Error bars: SD.

Astroglial differentiation requires concerted signaling from BMP2/4 and other signaling pathways [12], [13], therefore terminally differentiated astrocytes are most efficiently derived in vitro by exposure of NSCs to fetal calf serum (FCS) [5], [7]. Indeed, when self-renewing NSC culture medium was supplemented with 10% FCS, both non-irradiated and irradiated NSCs rapidly differentiated into mature astrocytes and strongly expressed the typical marker GFAP (Fig. 3B). This terminal differentiation was however maintained as long as cells were continuously exposed to growth factor-providing FCS, since serum-derived astrocytes readily reverted their fate to self-renewing NSC when switched back to the NSC culture medium, as determined by reduced *GFAP* levels and restored expression of *Nestin*, DDR gene *ATM* and proliferation marker *Ki67* (Fig. 3C).

The above results imply that NSC culture medium is incompatible to maintaining differentiation and its self-renewal impact can only be efficiently counteracted by the plethora of growth factors present in FCS. Therefore, self-renewing NSCs were irradiated and afterwards subjected to FCS treatment in order to provide them with appropriate culture conditions for astroglial differentiation. Remarkably, this approach significantly suppressed apoptosis following DNA damage, particularly when implemented early on, as compared to unmodified self-renewal conditions (Fig. 2E).

Thus, the delayed apoptosis observed in irradiated NSC cultures is likely to be independent of DNA damage *per se*, and instead seems to originate from the incompatibility of the self-renewal culture conditions for senescent and differentiating NSCs. Indeed, irradiation experiments in vitro do not affect the self-renewal “niche”, while it is likely to be different in an irradiated brain. This potentially intricate niche effect on NSCs viability after in vivo irradiation could account for inefficiency of caspase inhibitors to prevent radiation-induced apoptosis [14] and, on the other hand, increased survival of p53-deficient neural progenitors [15]. Therefore, stem cell niche effects and niche signaling should always be taken into account during irradiation studies on somatic stem cells.
